This article has been retracted.

# lncRNA CCAT1 promotes cell proliferation, migration, and invasion by down-regulation of miR-143 in FTC-133 thyroid carcinoma cell line

**DOI:** 10.1590/1414-431X20187046

**Published:** 2018-05-21

**Authors:** Tianzheng Yang, Hongyan Zhai, Ruihong Yan, Zhenhu Zhou, Lei Gao, Luqing Wang

**Affiliations:** 1 Department of Nuclear Medicine, Liaocheng People's Hospital, Liaocheng, Shandong, China; 2 Department of Radioimmunoassay, Liaocheng People's Hospital, Liaocheng, Shandong, China

**Keywords:** Thyroid cancer, CCAT1, miR-143, VEGF, PI3K/AKT pathway, MAPK pathway

## Abstract

Thyroid cancer is a common malignant tumor. Long non-coding RNA colon cancer-associated transcript 1 (lncRNA CCAT1) is highly expressed in many cancers; however, the molecular mechanism of CCAT1 in thyroid cancer remains unclear. Hence, this study aimed to investigate the effect of CCAT1 on human thyroid cancer cell line FTC-133. FTC-133 cells were transfected with CCAT1 expressing vector, CCAT1 shRNA, miR-143 mimic, and miR-143 inhibitor, respectively. After different treatments, cell viability, proliferation, migration, invasion, and apoptosis were measured. Moreover, the regulatory relationship of CCAT1 and miR-143, as well as miR-143 and VEGF were tested using dual-luciferase reporter assay. The relative expressions of CCAT1, miR-143, and VEGF were tested by qRT-PCR. The expressions of apoptosis-related factors and corresponding proteins in PI3K/AKT and MAPK pathways were analyzed using western blot analysis. The results suggested that CCAT1 was up-regulated in the FTC-133 cells. CCAT1 suppression decreased FTC-133 cell viability, proliferation, migration, invasion, and miR-143 expression, while it increased apoptosis and VEGF expression. CCAT1 might act as a competing endogenous RNA (ceRNA) for miR-143. Moreover, CCAT1 activated PI3K/AKT and MAPK signaling pathways through inhibition of miR-143. This study demonstrated that CCAT1 exhibited pro-proliferative and pro-metastasis functions on FTC-133 cells and activated PI3K/AKT and MAPK signaling pathways via down-regulation of miR-143. These findings will provide a possible target for clinical treatment of thyroid cancer.

## Introduction

Thyroid cancer is a common endocrine system malignant tumor, accounting for about 3% of all malignant tumors (1). It can be divided into two types: differentiated and undifferentiated (2). The five-year survival rate of differentiated thyroid cancer could reach 90%, but for the undifferentiated type, it is less than 10% (3). Over the past few decades, the incidence of thyroid cancer has been rising globally. Although this disease has improved with early diagnosis and treatment, the mortality rate has not declined (4). Hence, it is necessary to study the pathogenesis and regulatory mechanisms of thyroid cancer in order to effectively reduce mortality and improve clinical treatment.

With the rapid development of tumor molecular biology, many researchers have studied tumors using modern molecular technology. The findings show that tumor development involves a series of key molecules, such as cancer stem cells, long non-coding RNAs (lncRNAs), and microRNAs (miRNAs) (5 [Bibr B06]–7). These molecules are important for almost all cancers and are responsible for the modulation of the tumor microenvironment in malignant processes (7).

lncRNAs are a class of conserved non-coding RNA in eukaryotic cells with a length longer than 200 nt (8). Accumulating evidence suggests that a number of lncRNAs play important roles in the development of many cancers (9,10). For example, Tuo et al. reported that lncRNA UCA1 was up-regulated and could regulate cell proliferation and apoptosis in breast cancer by down-regulation of miR-143 (9). lncRNA GAS5 is low-expressed in lung cancer tissues and regulates cell proliferation and apoptosis by activating p53 and E2F1 signaling pathways (10). In addition, some lncRNA expressions could be used as markers for cancer diagnosis (11); for example, lncRNA PVT1 is an independent risk factor for hepatocellular carcinoma (HCC) recurrence (12). Furthermore, lncRNA colon cancer-associated transcript 1 (CCAT1) was first discovered in 2012 (13) and is highly expressed in many cancers, including gastric cancer, colon cancer, and HCC (14–16). Meanwhile, CCAT1 promotes proliferation, migration, and invasion of cancer cells inducing tumorigenesis and metastasis process. Moreover, Deng et al. (15) showed that CCAT1 boosts HCC progression via functioning as a let-7 sponge. However, the regulation and molecular mechanism of CCAT1 in the thyroid cancer remain unclear.

miRNAs are widely distributed in eukaryotes and can participate in many physiological processes, including proliferation, apoptosis, and differentiation of biological cells (5). In previous studies, miR-143 was found to be highly expressed in several cancers and was mainly identified as tumor suppressor by inhibiting tumor growth (17,18). Only one study reported that miR-143 expression was decreased in thyroid cancer and B-cell malignancies (18).

Therefore, we aimed to explore the molecular mechanism of lncRNA CCAT1 to reveal its potential in thyroid cancer therapy by focusing on the regulation between CCAT1 and miR-143.

## Material and Methods

### Cell culture

Human follicular thyroid carcinoma cell line FTC-133 (BNCC337959) and human thyroid normal cell line Nthy-ori 3–1 (BNCC340487) were purchased from BeNa Culture Collection (BNCC; China). The cells were cultured in 90% Dulbecco's Modified Eagle's Medium (DMEM; Solarbio, China) supplemented with 100 U/mL penicillin, 100 mg/mL streptomycin, and 10% heat-inactivated fetal bovine serum (FBS; all from Sigma-Aldrich, USA), and incubated in a humid atmosphere containing 5% CO_2_ at 37°C.

### Cell transfection

In order to test CCAT1 expression, short-hairpin RNA (shRNA) directed against human lncRNA CCAT1 was ligated into the U6/GFP/Neo plasmid (GenePharma, China) to become sh-CCAT1. The full-length CCAT1 sequence was constructed in pEX-2, and was called pEX-CCAT1. The plasmid carrying a non-targeting sequence was used as a negative control (NC) of sh-CCAT1 that was referred to as sh-NC. miR-143 mimic, inhibitor, and their respective NCs were synthesized and transfected into FTC-133 cells in this study (GenePharma). Following the manufacturer's instructions, cell transfection was performed using Lipofectamine^TM^ 3000 reagent (Thermo Fisher Scientific, USA). The stably transfected cells were selected by the culture medium containing 0.5 mg/mL G418 (Sigma-Aldrich, USA). After approximately 4 weeks, G418-resistant FTC-133 cells were established and collected for the subsequent experiments.

### Cell viability assay

FTC-133 cells were seeded in 96-well plates with 2×10^3^ cells/well and assessed by Cell Counting Kit-8 (CCK-8; Dojindo Molecular Technologies, USA). Briefly, 10 μL of CCK-8 solution was added to each well, and the cultures were then incubated for 1 h at 37°C in humidified 95% air and 5% CO_2_. The experiment was repeated three times. Absorbance was measured at 450 nm using a Microplate Reader (Bio-Rad, Hercules, USA).

### Cell proliferation assay

FTC-133 cells were seeded in 96-well plates with 2×10^3^ cells/well. Cell proliferation was evaluated using BrdU Cell Proliferation Assay Kit (Sigma-Aldrich) following the manufacturer's instructions. In brief, BrdU was added to each well, and cultures were incubated for 40 min at 37°C. Cells were then washed in phosphate buffered saline (PBS) twice and fixed with methanol for 10 min. Each experiment was repeated at least three times independently. Absorbance was measured at 450 nm using a Microplate Reader (Bio-Rad).

### Cell migration and invasion assay

Cell migration was determined using a modified two-chamber method with a pore size of 8-μm membranes. FTC-133 cells (2×10^4^ /ml) were suspended in 100 μl of serum-free DMEM medium and seeded on the upper compartment of 24-well Transwell culture chamber (Millipore, USA). DMEM (500 μL) medium including 10% fetal bovine serum (FBS; Sijiqing, China) was added to the lower compartment. After incubation for 24 h at 37°C in 5% CO_2_ atmosphere, all cells were fixed with 95% ethanol for 30 min. Non-traversed cells were removed from the upper surface of the filter carefully with a cotton swab; the traversed cells on the lower side of the filter were stained with 0.5% crystal violet (Solarbio, China) for 30 min and counted under a microscope (Leica Microsystems, Germany). The experiment was repeated three times.

Cell invasion was measured using 24-well Millicell¯ Hanging Cell Culture Inserts with 8-μm PET membranes (Millipore). FTC-133 cells (2×10^4^/mL) in 200 μL serum-free DMEM medium were plated onto BD BioCoat^TM^ Matrigel^TM^ Invasion Chamber (BD Biosciences, USA), while DMEM medium containing 10% FBS was added to the lower chamber. After processing the invasion chambers for 48 h at 37°C (5% CO_2_) in accordance with the manufacturer's protocol, the non-invading cells were removed with a cotton swab. The invading cells were fixed in 100% methanol for 30 min, stained with 0.5% crystal violet solution for 30 min, and then counted microscopically. The experiment was repeated three times.

### Apoptosis assay

Apoptotic assays were performed using Annexin V-FITC/PI Apoptosis Detection Kit (Sigma-Aldrich). In brief, stable FTC-133 cells (2×10^4^ /mL) were washed in cold PBS three times and stained in 200 µL of binding buffer including 10 µL Annexin V-FITC and 5 µL of PI in the presence of 50 μg/mL RNase A (Sigma-Aldrich), and then incubated for 1 h at room temperature in the dark. Flow cytometry analysis was done using a FACScan (Beckman Coulter, USA). The data were analyzed by using FlowJo software (Treestar, Inc., USA).

### Dual-luciferase reporter assay

The fragment from CCAT1 was amplified by PCR and then cloned into a pmirGLO dual-luciferase miRNA Target Expression Vector (Promega, USA). Then, miR-143 mimics were individually co-transfected with the reporter vector CCAT1-wild-type (CCAT1-wt) or CCAT1-mutated-type (CCAT1-mt) into FTC-133 cells. The fragment from VEGF 3′UTR was amplified by PCR and then cloned into a pmirGLO dual-luciferase miRNA Target Expression Vector (Promega). miR-143 mimics were individually co-transfected with the reporter vector VEGF 3′UTR-wild-type (VEGF 3′UTR-wt) or VEGF 3′UTR-mutated-type (VEGF 3′UTR-mt) into FTC-133 cells. Dual-luciferase¯ Reporter Assay System Protocol (Promega) was used to measure the luciferase activity after 48 h of cell transfection and collection. The experiment was repeated three times independently.

### Quantitative real-time polymerase chain reaction (qRT-PCR)

According to the manufacturer's instructions, total RNA was extracted from FTC-133 cells using Trizol reagent (Life Technologies Corporation, USA). The expression level of CCAT1 was tested using One Step SYBR¯ PrimeScript¯ PLUS RT-RNA PCR Kit (TaKaRa Biotechnology, China). The Taqman MicroRNA Reverse Transcription Kit and Taqman Universal Master Mix II (both from Applied Biosystems, USA) were used to detect the level of miR-143 expression. The GAPDH and U6 were used in this study for normalizing CCAT1 and miR-143 levels. The sequences of qRT-PCR primers were as follows: lncRNA CCAT1, 5′-AGAAACACTATCACCTACGC-3′ (Forward) and 5′-CTTAACAGGGCATTGCTAATCT-3′ (Reverse); miR-143, 5′-AAGCTTAAGGTCAAGGTTTGGTCCT-3 (Forward) and 5′-CTCGAGTGCTAAGATGGACACACTGG-3′ (Reverse); U6, 5′-CGCTTCGGCAGCACATATACTA-3′ (Forward) and 5′-CGCTTCACGAATTTGCGTGTCA-3′ (Reverse); GAPDH, 5′-TGTTGCCATCAATGACCCCTT-3′ (Forward) and 5′-CTCCACGACGTACTCAGCG-3′ (Reverse); sh-CCAT1, 5′-CCTGGCCCTCTCATCAGAGACTTGACTTA-3′; miR-143 mimic, 5′-GGUGCAGUGCUGCAUCUCUGGU-3′ (mimics sense) and 5′-CAGAGAUGCAGCACUGCACCUU-3′ (mimics antisense); and miR-143 inhibitor, 5′-ACCAGAGAUGCAGCACUGCACC-3′. Fold changes were calculated by the relative quantification (2^−ΔΔCt^) method (19).

### Western blot analysis

RIPA lysis buffer (Beyotime Biotechnology, China) supplemented with protease inhibitors (Roche, China) was used to extract the proteins for western blot analysis. Proteins were quantified using the BCA™ Protein Assay Kit (Pierce, Appleton, USA) following the manufacturer's protocol. Then, proteins (30 μg/sample) were loaded, electrophoresed by 10% sodium dodecyl sulfate-polyacrylamide gel electrophoresis (SDS-PAGE), and transferred to the polyvinylidene difluoride (PVDF) membranes. The primary antibody of VEGFA (ab46154), Bcl-2 (ab32124), Bax (ab32503), pro-caspase-3 (ab32499), cleaved-caspase-3 (ab2302), pro-caspase-9 (ab135544), cleaved-caspase-9 (ab2324), PI3K p85 (ab191606), p-P13K p85 (ab182651), AKT (ab8805), p-AKT (ab38449), MAPKAP Kinase 2 (ab131531), p-MAPKAP Kinase 2 (ab131504), and GAPDH (ab9485) were obtained from Abcam (China), prepared in 5% blocking buffer at a dilution of 1:1000, incubated with the membrane for 2 h at 4°C, washed twice in PBS, and then cultivated with secondary antibody (1:1000) marked by horseradish peroxidase for 2 h at room temperature. Immobilon Western chemiluminescent HRP substrate (200 μL; Millipore) was added to cover the membrane surface, the signals were captured, and the intensity of the bands was quantified using Image Lab™ software (Bio-Rad).

### Statistical analysis

The results are reported as means±SD. Statistical analyses were performed using SPSS 19.0 statistical software (IBM Corporation, USA). The P-values were calculated using a one-way analysis of variance (ANOVA). P*<*0.05 indicated a statistically significant result.

## Results

### CCAT1 overexpression enhanced cell viability, proliferation, migration, and invasion in FTC-133 cells

In order to assess the effect of CCAT1 on thyroid carcinoma cells, we first detected the expression level of CCAT1 in different cell lines using qRT-PCR, and found that CCAT1 was up-regulated in thyroid carcinoma cell line FTC-133 compared with human thyroid normal cell line Nthy-ori 3–1 (P<0.01, Figure 1A). The transfection efficiency of CCAT1 overexpression and suppression were examined in FTC-133 cells. As shown in Figure 1B and C, CCAT1 expression was significantly down-regulated in the sh-CCAT1 group and up-regulated in the pEX-CCAT1 group (both P<0.01). The results of CCK-8, BrdU, Transwell, and invasion assay (Figure 2A and D) showed that cell viability, proliferation, migration, and invasion were all increased when CCAT1 was overexpressed (all P<0.05). However, suppression of CCAT1 displayed the opposite results; that is, cell viability, proliferation, migration, and invasion were greatly reduced (all P<0.05). Subsequently, apoptosis and the expressions of apoptosis-related proteins were detected using flow cytometry analysis and western blot, respectively. The results suggested that apoptosis was significantly elevated by CCAT1 knockdown (P<0.001). The expression of Bcl-2 was down-regulated and Bax, cleaved-caspase-3, and cleaved-caspase-9 expressions were up-regulated in sh-CCAT1 group (Figure 2E and F). Moreover, CCAT1 overexpression had little effect on apoptosis.

**Figure 1.** Expression of CCAT1 in FTC-133 cells. Cells were transfected with CCAT1 expressing vector or CCAT1 shRNA. *A*, The mRNA level of CCAT1 was detected using qRT-PCR in Nthy-ori 3–1 cells and FTC-133 cells. *B* and *C*, The expression level of CCAT1 suppression and overexpression were tested by using qRT-PCR in FTC-133 cells. NC: negative control. Data are reported as means±SD. **P<0.01 (ANOVA).

**Figure 2.** CCAT1 increased cell viability, proliferation, migration, and invasion in FTC-133 cells. Cells were transfected with CCAT1 expressing vector or CCAT1 shRNA. *A* to *E*, Cell viability, proliferation, migration, invasion, and apoptosis were measured using CCK-8, BrdU assay, Transwell assay, invasion assay, and flow cytometry analysis, respectively. *F*, The expressions of apoptosis-related proteins were detected using western blot analysis. NC: negative control. Data are reported as means±SD. *P<0.05; ***P<0.001 (ANOVA).

### CCAT1 overexpression promoted vascular endothelial growth factor (VEGF) expression in FTC-133 cells via down-regulation of miR-143

The regulatory relationship between CCAT1 and miR-143 was detected using qRT-PCR and dual-luciferase reporter assay. Thus, the expressing vector and shRNA of CCAT1 were transfected into FTC-133 cells to overexpress and silence CCAT1 expression, respectively. The expression of miR-143 was clearly up-regulated by CCAT1 suppression and down-regulated by CCAT1 overexpression in FTC-133 cells (P<0.05 or P<0.01; Figure 3A). Figure 3B showed that CCAT1 had binding sites for miR-143, which might better explain the negative regulatory relationship between CCAT1 and miR-143. Therefore, we suspected that CCAT1 might be working as a competitive endogenous RNA (ceRNA) for miR-143. To verify this hypothesis, dual-luciferase reporter assay was performed. The relative luciferase activity in FTC-133 cells that were co-transfected with CCAT1-wt and miR-143 mimic was lower than the cells co-transfected with CCAT1-mt and NC (P<0.05; Figure 3C). Shown in Figure 3D and E, the results of qRT-PCR and western blot displayed that CCAT1 knockdown decreased the expression of VEGF, while the opposite results were observed in pEX-CCAT1 group (P<0.05 or P<0.01). To further explore the relationship between miR-143 and VEGF in FTC-133 cells, we analyzed VEGF expression in cells transfected with miR-143 mimic or inhibitor. As shown in Figure 3F, efficiency of miR-143 up-regulation and inhibition was confirmed by using qRT-PCR. Figure 3G and H suggested that the mRNA and protein levels of VEGF were reduced in miR-143 mimic-treated cells, while miR-143 inhibitor up-regulated the expression of VEGF (P<0.05 or P<0.01). As shown in Figure 3I, there was a binding site for miR-143 in VEGF. The relative luciferase activity in FTC-133 cells co-transfected with VEGF 3UTR-wt and miR-143 mimic was lower than cells co-transfected with VEGF 3UTR-mt and NC (P<0.05, Figure 3J). Therefore, miR-143 and VEGF exhibited the negative regulatory relationship, which explained the positive regulation of CCAT1 on VEGF.

**Figure 3.** CCAT1 promoted the up-regulation of VEGF via inhibition of miR-143. FTC-133 cells were transfected with CCAT1 expressing vector, CCAT1 shRNA, miR-143 mimic, or miR-143 inhibitor. *A*, mRNA expression of miR-143 was detected in FTC-133 cells using qRT-PCR. *B*, The predicated miR-143 binding site of CCAT1 (CCAT1-wt) and the designed CCAT1-mt are indicated. *C*, The binding relationship between CCAT1 and miR-143 was assessed using dual-luciferase reporter assay. *D*, mRNA levels of VEGF in FTC-133 cells were detected using qRT-PCR. *E*, The protein level of VEGF with sh-CCAT1 or pEX-CCAT1 was analyzed using western blot analysis. *F*, *G*, mRNA levels of miR-143 and VEGF with miR-143 mimic or inhibitor were tested using qRT-PCR. *H*, The protein level of VEGF with miR-143 mimic or inhibitor were detected using western blot analysis. *I*, The predicted miR-143 binding site of VEGF 3′UTR (VEGF 3′UTR-wt) and the designed VEGF 3′UTR-mt are indicated. *J*, The binding relationship between miR-143 and VEGF 3′UTR was assessed using dual-luciferase reporter assay. NC: negative control. Data are reported as means±SD. *P<0.05; **P<0.01 (ANOVA).

### CCAT1 overexpression increased cell viability, proliferation, migration, and invasion in FTC-133 cells by down-regulating miR-143 expression

The effects of CCAT1 in combination with miR-143 were further studied on FTC-133 cells. CCAT1 overexpression plus miR-143 overexpression decreased cell viability and proliferation relative to only CCAT1 overexpression (both P<0.05; Figure 4A to D). Cell viability and proliferation were increased after CCAT1 suppression plus miR-143 knockdown relative to only CCAT1 suppression (both P<0.05). Similarly, miR-143 overexpression inhibited the increases of cell migration and invasion induced by CCAT1 overexpression; on the contrary, miR-143 knockdown enhanced the reduction of migration and invasion induced by CCAT1 suppression (all P<0.05; Figure 5A to D). In addition, we also detected expressions of apoptosis and apoptosis-related proteins by the treatments of miR-143 silence combined with CCAT1 suppression. As shown in Figure 5E and F, apoptosis, Bax, and cleaved caspase-3/9 expressions were significantly reduced; Bcl-2 expression was simultaneously increased in sh-CCAT1+miR-143 inhibitor group compared with sh-CCAT1+NC group (P<0.05).

**Figure 4.** CCAT1 enhanced cell viability and proliferation via the inhibition of miR-143. FTC-133 cells were transfected with CCAT1 expressing vector, CCAT1 shRNA, miR-143 mimic, or miR-143 inhibitor. *A* and *B*, Cell viability, and *C* and *D*, proliferation were measured in FTC-133 cells using CCK-8 and BrdU assay, respectively. NC: negative control. Data are reported as means±SD. *P<0.05 (ANOVA).

**Figure 5.** CCAT1 enhanced cell migration and invasion via the inhibition of miR-143. FTC-133 cells were transfected with CCAT1 expressing vector, CCAT1 shRNA, miR-143 mimic, or miR-143 inhibitor. *A* and *B*, Cell migration, *C* and *D*, invasion, and (*E*) apoptosis were measured in FTC cells using Transwell assay, invasion assay, and flow cytometry analysis, respectively. *F*, The expressions of apoptosis-related proteins were detected using western blot analysis. NC: negative control. Data are reported as means±SD. *P<0.05, ***P<0.001 (ANOVA).

### CCAT1 overexpression activated PI3K/AKT and MAPK signaling pathways via down-regulation of miR-143

The expressions of the proteins associated with PI3K/AKT and MAPK signaling pathways were assessed using western blot analysis. The results (Figure 6A and B) displayed that the levels of p-P13K p85, p-AKT, and p-MAPKAP kinase 2 were all obviously up-regulated after CCAT1 overexpression, and then miR-143 overexpression inhibited these increases. Conversely, CCAT1 knockdown down-regulated p-P13K, p85, p-AKT, and p-MAPKAP Kinase 2 expressions, while their expressions were further increased after miR-143 suppression.

**Figure 6.** CCAT1 activated PI3K/AKT and MAPK signaling pathways via the inhibition of miR-143. FTC-133 cells were transfected with CCAT1 expressing vector, CCAT1 shRNA, miR-143 mimic, or miR-143 inhibitor. The expressions of the main factors in *A*, PI3K/AKT and *B*, MAPK signaling pathways were analyzed in FTC-133 cells using western blot analysis. NC: negative control.

## Discussion

Thyroid cancer is characterized by high morbidity and rapid growth in China (20). lncRNAs can participate in the regulation of cell proliferation, migration, and apoptosis by controlling the expression of downstream miRNAs (21,17). Therefore, we studied the regulatory mechanism of lncRNA CCAT1 on thyroid cancer cell line FTC-133. CCAT1 was closely related with colon cancer genesis, and down-regulation of miR-143 was a well-known potential marker for colon cancer and played an important role in carcinogenesis (22,23). Therefore, we analyzed the binding site of CCAT1 and miR-143. As CCAT1 was up-regulated in FTC-133 cells, the regulatory relationship of CCAT1 and miR-143 in FTC-133 cells were analyzed and the effects of CCAT1-miR-143 axis on FTC-133 cells were also explored. Furthermore, the mechanism of CCAT1 was investigated by detecting activations of PI3K/AKT and MAPK signaling pathways after altering expressions of CCAT1 and miR-143.

Our study suggested that CCAT1 might act as a competing endogenous RNA (ceRNA) for miR-143. CCAT1 overexpression up-regulated miR-143-mediated VEGF expression, indicating that CCAT1 might promote angiogenesis in thyroid carcinoma. CCAT1 overexpression enhanced cell viability, proliferation, migration, and invasion, as well as reduced apoptosis by down-regulation of miR-143. In addition, we also found that CCAT1 activated PI3K/AKT and MAPK signaling pathways by inhibiting miR-143 expression.

lncRNA CCAT1 is a non-coding RNA with the length of 2628 nt and originally found in colon cancer (13). A large number of studies have shown that knockdown of CCAT1 significantly inhibited cell proliferation and migration and promoted apoptosis in many cancers, including glioma (21), prostate cancer (24), and HCC (15), suggesting that CCAT1 was an oncogene. In our study, we first found that CCAT1 was overexpressed in FTC-133 cells. Further results showed that CCAT1 overexpression increased cell viability, proliferation, migration, and invasion, but obviously reduced apoptosis of FTC-133 cells. These findings were consistent with previous studies (15,21,24), implying that CCAT1 could promote cancer growth in FTC-133 cells.

miR-143 has been reported to decrease prostate cancer cells' proliferation and migration (25). Moreover, a previous study reported that miR-143 is down-regulated in thyroid cancer (18). However, the results of our study revealed that overexpression of miR-143 inhibited increases of cell viability, proliferation, migration, invasion, and the reduction of apoptosis in FTC-133 cells. Therefore, we speculated that miR-143 was a tumor suppressor for thyroid cancer and upstream regulated CCAT1. Recent studies have demonstrated that lncRNAs function as ceRNA by sponging miRNAs to regulate gene expression at a post-transcriptional level (26). For instance, CCAT1 could competitively bind miR-218-5p through intracellular “sponge-like” adsorption and promote the expression of target genes, leading to the proliferation of bladder cancer cells and invasion of blood vessels (27). Thus, we explored the regulatory relationship between CCAT1 and miR-143 in this study. Firstly, we found that CCAT1 overexpression down-regulated the expression of miR-143. There was a binding site of miR-143 in the sequence of CCAT1. Then, relative luciferase activity was lower in cells co-transfected with CCAT1-wt and miR-143 mimic. Considering the context, we deduced that CCAT1 could act as a molecular sponge in regulating the biological functions of miR-143. In addition, VEGF is an important factor in mediating angiogenesis, which can promote the mitosis of vascular endothelial cells and the growth of tumor blood vessels (28 [Bibr B29]). Related evidence has shown that lncRNAs and miRNAs regulate the expression of VEGF in cancers (28–30). In the current study, we found that CCAT1 positively and miR-143 negatively regulated VEGF expression. Further, the mRNA and protein level of VEGF were increased with CCAT1 overexpression or miR-143 suppression. Importantly, there was a binding site of VEGF in the sequence of miR-143 and the dual-luciferase reporter assay further confirmed their positive regulatory relationship. Therefore, VEGF also plays an important role in the study of thyroid cancer.

Pagliuca et al. (31) reported that Kirsten rat sarcoma 2 viral oncogene homolog (KRAS) and v-Raf murine sarcoma viral oncogene homolog B1 (BRAF) were targeted by miR-143. The reduction of the expressions of these proteins affected cell signaling pathways involved in transformation. Moreover, the primary mediators of miR-143 in inhibiting tumors are genes belonging to the growth factor receptor-mitogen-activated protein kinase (MAPK) network. Wang et al. (32) showed that miR-143 overexpression inhibited PI3K/AKT signaling pathway in glioma and other RAS-driven cancers. Hence, we focused on P13K/AKT and MAPK pathways to explain the effect of CCAT1 on FTC-133 cells. P13K/AKT pathway is the central regulator of cell growth, proliferation, apoptosis, and metabolism (33). MAPK is a primary pathway for signal transduction of vascular endothelial cells (34 [Bibr B35]). Recently, extensive research has shown that the activated P13K/AKT and MAPK signaling pathways could promote tumor cell proliferation, invasion, and migration and reduce apoptosis (34–36). Our results suggested that CCAT1 overexpression increased the expression of proteins associated with these pathways, whereas miR-143 overexpression inhibited these effects. CCAT1 could activate PI3K/AKT and MAPK signaling pathways by inhibiting miR-143 expression.

In summary, our study demonstrated that CCAT1 exhibited a cancer-promoting function potentially via down-regulation of miR-143 and activation of PI3K/AKT and MAPK signal pathways in FTC-133 cells. Hence, this study might provide a basis for further study of the mechanism of lncRNA CCAT1 and a possible target for the clinical treatment of thyroid cancer.
